# Study on the Rural Revitalization and Urban-Rural Integration Efficiency in Anhui Province Based on Game Cross-Efficiency DEA Model

**DOI:** 10.1155/2022/7373435

**Published:** 2022-04-13

**Authors:** Shanhui Sun, Ni-Ni Zhang, Jia-Bao Liu

**Affiliations:** ^1^College of Mathematics and Statistics, Suzhou University, Suzhou, Anhui 234000, China; ^2^School of Management, Suzhou University, Suzhou, Anhui 234000, China; ^3^School of Mathematics and Physics, Anhui Jianzhu University, Hefei 230601, China

## Abstract

By taking the 16 cities in Anhui Province for evaluation, the main influencing factors and indicator system for integrated urban-rural development in the new era were explored, to build the BCC model, cross-efficiency model, and game cross-efficiency model of DEA. The above models were applied for empirical analysis and comparative study on the rural revitalization and urban-rural integration efficiency in Anhui Province, to summarize the conclusions efficiency and give suggestions based on the above calculations.

## 1. Introduction

City and countryside serve as two important constituents in social life, and the whole society's prosperity and development rest upon the sustainable development of these two parts. Rural revitalization and urban-rural integration supplement each other, so the study on their intrinsic logical relation shall be aimed at the complexity and dynamics of urban-rural regional system and exploring the construction plan, mode, and scientific method for eliminating urban-rural gap [1].

In September 2018, the issuance of the Plan for the Rural Revitalization Strategy (2018–2022) marked that rural revitalization stepped into the specific implementation stage and became the focus of attention of domestic scholars. Chinese government provides its scholars with the research direction of rural revitalization through land reform, socialism market system reform, and development of the beautiful village and modern agriculture [2]. Rural revitalization aims at establishing the system and mechanism for integrated urban-rural development and constructing the comprehensive development system for rural area, including the reformation, reconstruction, and innovation according to the requirements of thriving enterprises, pleasant living environment, convenance, civilized and effective governance, and prosperity.

Therefore, the urgent problem for rural revitalization is to objectively recognize the differences between urban living quality and rural living quality and identify the urban-rural integration degree, which is of important guiding significance to improving the living quality in urban and rural areas and promoting the formulation of the policies for integrated urban-rural development [3].

## 2. Current Situations of Domestic and Overseas Research

Along with the development of globalization and urbanization, different countries and regions are all faced with various problems and conflicts. Foreign countries mainly took the following policies for rural revitalization: New Countryside Movement in South Korea, Comprehensive Village and Town Construction Demonstration Project in Japan, European Common Agricultural Policy (2014–2020), Japan's agricultural support policy and the study on rural economic development in Italy.

Rural-urban fringe zone refers to the transitional area combining the factors. As the border of urban expansion and the reserved land in rural area, rural-urban fringe zone has to solve the problem of urban-rural land use, which results in traffic jam, environmental pollution, and living quality degradation. Therefore, in order to effectively present the microdynamic development of the marginal area between city and countryside, it is necessary to guide the effective use of land. In Herberholz's opinion, urban-rural relationship is fundamental in the social development of human beings and also important to be solved in regional development [4]. Lysgard believes that theoretically, there are three main trends in the development of rural-urban relations: urban orientation, urban-rural interaction, and rural orientation [5]. Schmidt and Piloyan considered that the land element in the transitional area is one of the key points of the research by foreign scholars [6, 7]. Hachem successively proposed the concept of mixed community, which was strongly recommended and applied in the construction of modern integrated urban-rural development. It is used to promote the local economy by encouraging unity, supporting network, enhancing safety, and creating job opportunities [8].

The urban-rural dual structure gives priority to urban development, and labor force, resources, and capital are input for urban construction, resulting in a series of problems, such as village hollowing, environmental pollution, weakening of agriculture. Urban and rural areas are an interactive organism, and they are contradictory, coordinated, integrated, and equivalent, so rural revitalization is the only road for urban-rural integration.

Zheng et al. believe that pluralities of fields are covered for implementing rural revitalization strategy, including social governance, industrial development, and rural civilization, and all stakeholders shall develop top-level policy design for the rural revitalization strategy. We can really promote the integrated urban-rural development only by changing the development concept, allocating production factors efficiently, and optimizing the economic structure [9]. Li and Bo consider that it is necessary to put forward the overall plan for “development in five areas,” seeking the inherent thought train for realizing the urban-rural integration [10]. Zhang and Zhao elaborate the basic frame of urban-rural integration from the consistency among objectives, essence, and space of rural revitalization strategy and integrated urban-rural development and put forth the result-based common development [11]. Li believes that the key to rural revitalization lies in urban-rural integration which is the objective law and also the effect form coping with risks and crises. Either-or thinking is not applicable to rural revitalization and urbanization; overall planning must be made for development in the process of promoting the rural revitalization strategy to realize integrated urban-rural development [12].

## 3. Research Methods, Data Source, and Index Construction

### 3.1. Research Methods

It analyzes the process and effect of rural revitalization and integrated urban-rural development by comprehensively applying the theory and method of system science and management. It analyzes indexes systemically with methods of statistics and operational research and builds scientific evaluation models and path selection models with data mining and mathematical modeling to provide a theoretical basis for path selection of rural revitalization and integrated urban-rural development.

### 3.2. Data Source and Index Construction

In this paper, the data are mainly from Anhui Statistical Yearbook, and the urban-rural integration is comprehensive and analyzed from the spatial arrangement, industry configuration, income gap, public service, and ecological environment. It makes crossover analysis on rural revitalization and urban-rural integration and finds their intersection combining with the statistical index of Anhui Statistical Yearbook. The analysis is detailed in the following Table 1.

In the table, *X*1 indicates the ratio between nonagricultural workers and agricultural workers, *X*2 refers to the ratio between nonagricultural production value and agricultural production value, *X*3 means the ratio of hospital bed, *X*4 refers to the ratio of the number of days with the air quality of and above Level II between urban and rural areas, *X*5 refers to the ratio of subsistence allowances amount per capita, *X*6 indicates the ratio of the number of students enrolled in middle schools, *X*7 means the green coverage ratio in built-up areas, *X*8 refers to the sewage treatment rate, and *X*9 refers to the ratio of disposable income. Moreover, *Y*1 is the variable and is expressed by the urbanization rate of residents [13].

## 4. Construction of Game Cross-Efficiency Model

First, it finds out the major influencing factors by factor analysis and carries out factor analysis for the original variables by data mining [14]. Second, it evaluates the efficiency by inputting three kinds of models of data envelopment analysis.

### 4.1. Principal Component Analysis

It means to classify variables based on the relevance of variables in systems and take the classified variables as the principal component to show the main system information with less principal component. *n* decision bodies and *p* evaluation indexes are provided, and the original data are

(1) $$\begin{array}{c} X=\left(\begin{array}{cccc} x_{11} & x_{12} & ... & x_{1p}\\ x_{21} & x_{22} & ... & x_{2p}\\ ... & ... & ... & ...\\ x_{n1} & x_{n2} & ... & x_{np} \end{array}\right). \end{array}$$

The correlation factor matrix is calculated as

(2) $$\begin{array}{c} R=\left(\begin{array}{cccc} r_{11} & r_{12} & ... & r_{1p}\\ r_{21} & r_{22} & ... & r_{2p}\\ ... & ... & ... & ...\\ r_{n1} & r_{n2} & ... & r_{np} \end{array}\right), \end{array}$$

where *r*_*ij*_(*i*, *j*=1,2,…, *p*) is the correlation factor between the *i* th and the *j* th evaluation indexes.

(3) $$\begin{array}{c} r_{ij}=\frac{\sum_{k=1}^{n}\left(x_{ki}-\bar{x_{i}}\right)\left(x_{kj}-\bar{x_{j}}\right)}{\sqrt{\sum_{k=1}^{n}{\left(x_{ki}-\bar{x_{i}}\right)}^{2}\sum_{k=1}^{n}{\left(x_{kj}-\bar{x_{j}}\right)}^{2}}}, \end{array}$$

where

(4) $$\begin{array}{c} \bar{x_{i}}=\frac{1}{n}\sum_{k=1}^{n}x_{ki},\\ \bar{x_{j}}=\frac{1}{n}\sum_{k=1}^{n}x_{kj}. \end{array}$$

The eigenvalue and eigenvector of *R* are calculated. The equation |*λI* − *R*|=0 is solved to work out the eigenvalue *λ*_*i*_, the eigenvalue *λ*_*i*_ in order of size *λ*_1_ ≥ *λ*_2_ ≥ …≥*λ*_*p*_ ≥ 0 is arranged, the corresponding eigenvector $\overset{⟶}{e_{i}}$(*i*=1,2,…, *p*) is calculated; ∑_*j*=1_^*p*^*e*_*ij*_^2^=1, *e*_*ij*_ is the *j* th component of vector $\overset{⟶}{e_{i}}$.

The contribution rate is

(5) $$\begin{array}{c} \frac{\lambda_{i}}{\sum_{k=1}^{p}\lambda_{p}}\left(i=1,2,\ldots ,p\right). \end{array}$$

The accumulative contribution rate is

(6) $$\begin{array}{c} \frac{\sum_{k=1}^{i}\lambda_{k}}{\sum_{k=1}^{p}\lambda_{p}}\left(i=1,2,\ldots ,p\right). \end{array}$$

Generally, the eigenvalue of the principal component with the accumulative contribution rate of 85%–95% is used; *λ*_1_, *λ*_2_,…, *λ*_*m*_ are, respectively, the 1st, 2nd, and …, the *m*(*m* ≤ *p*)th principal component.

The principal component load is calculated as follows:

(7) $$\begin{array}{c} l_{kij}=p\left(z_{k},x_{ij}\right)=\sqrt{\lambda_{i}}e_{kij}, \end{array}$$

where *k*=1,2,…, *n*; *i*, *j*=1,2,…, *p*.

Principle component is extracted, the load *l*_*kij*_, (*k*=1,2,…, *n*;  *i*, *j*=1,2,…, *p*) of original variables *x*_*kj*_(*k*=1,2,…, *n*; *i*, *j*=1,2,…, *p*) on principle component *z*_*k*_(*k*=1,2,…, *n*) is determined, and the representation of principle component of original data is

(8) $$\begin{array}{c} Z=\left(\begin{array}{cccc} z_{11} & z_{12} & ... & z_{1m}\\ r_{21} & r_{22} & ... & r_{2m}\\ ... & ... & ... & ...\\ x_{n1} & x_{n2} & ... & x_{nm} \end{array}\right), \end{array}$$

where

(9) $$\begin{array}{c} z_{i1}=l_{1i_{1}}x_{i_{1}}+l_{1i_{2}}x_{i_{2}}+\ldots +l_{1i_{p}}x_{i_{p}}\\ z_{i2}=l_{2i_{1}}x_{i_{1}}+l_{2i_{2}}x_{i_{2}}+\ldots +l_{2i_{p}}x_{i_{p}}\\ \ldots \\ z_{im}=l_{mi_{1}}x_{i_{1}}+l_{mi_{2}}x_{i_{2}}+\ldots +l_{mi_{p}}x_{i_{p}}. \end{array}$$

### 4.2. Envelopment Analysis Model

When the scale benefit is changeable, Banker, Charnes, and Cooper propose to evaluate the BCC model for decision-making unit *U*_0_, and the oriented model is input in the type of

(10) $$\begin{array}{c} \min\left(\theta -\varepsilon \left(e^{T}s^{-}+e^{T}s^{+}\right)\right)\text{s.t.}\sum_{i=1}^{n}\left(x_{ij}\lambda_{i}\right)+s^{-}=\theta x_{0j},\;j=1,2,\ldots ,m,\\ \sum_{i=1}^{n}\left(y_{ir}\lambda_{j}\right)+s^{+}=\theta y_{0r},\;r=1,2,\ldots ,s,\\ \sum_{i=1}^{n}\lambda_{i}=1,\lambda_{j}\geq 0,s^{+}\geq 0,s^{-}\geq 0. \end{array}$$

*x*_*ij*_ and *y*_*ir*_ are the input and output factors, respectively, and *θ* is the effective value of *U*_0_.

If *θ*=1, *s*^+^=*s*^−^=1, *U*_0_ means DEA is effective; if *θ*=1, *s*^+^ ≠ 1 or *s*^−^ ≠ 1, *U*_0_ means weak DEA is effective; if *θ* < 1, *U*_0_ refers to non-DEA is effective.

### 4.3. Cross-Efficiency Evaluation

The linear programing (LP) type is as follows:

(11) $$\begin{array}{c} \max\sum_{r=1}^{s}u_{r}y_{rd}=\theta_{d}\\ \text{s.t.}\sum_{i=1}^{m}\omega_{i}x_{ij}-\sum_{r=1}^{s}u_{r}y_{rd}\geq 0,\;j=1,2,\ldots ,n,\\ \sum_{i=1}^{m}\omega_{i}x_{id}=1.\\ \omega_{i}\geq 0,\;i=1,2,\ldots ,m,\\ u_{r}\geq 0,\;r=1,2,\ldots ,s, \end{array}$$

We get a group of optimal weight value (multiplier) *ω*_1  *d*_^*∗*^,…, *ω*_*m*  *d*_^*∗*^, *μ*_1  *d*_^*∗*^,…, *μ*_*s*  *d*_^*∗*^ for each *DM*  *U*_*d*_(*d*=1,2,…, *n*) evaluation. The cross-efficiency of any *DM*  *U*_*j*_(*j*=1,2,…, *n*) can be expressed and calculated below with the weight chosen by DMU.

(12) $$\begin{array}{c} E_{dj}=\frac{\sum_{r=1}^{s}u_{rd}^{*}y_{rj}}{\sum_{i=1}^{m}\omega_{id}^{*}x_{ij}},\;d,j=1,2,\ldots ,n. \end{array}$$

As shown in Table 2, when we move along the line *d* in the cross-efficiency matrix *E*, each factor *E*_*dj*_ is the cross-efficiency of *DM*  *U*_*d*_ and *DM*  *U*_*j*_, and the main diagonal thereof is a special case for DMU self-evaluation [15].

Then, everyone averages the column of the cross-efficiency matrix in Table 1. The average value of all *E*_*dj*_(*j*=1,2,…, *n*) for *DM*  *U*_*j*_(*j*=1,2,…, *n*), is $\bar{E_{dj}}$, namely, $\bar{E_{dj}}=1/n\left(E_{1j}+E_{2j}+\ldots +E_{nj}\right)$.

### 4.4. Game Cross-Efficiency

During the calculation of game cross-efficiency, the efficiency of *U*_*d*_ is set as *α*_*d*_; the optimal weight on the premise of ensuring no reduced *α*_*d*_ to maximize the self-efficiency [16] is obtained. The game cross-efficiency is

(13) $$\begin{array}{c} \alpha_{dj}=\frac{\sum_{r=1}^{s}u_{rjd}y_{rj}}{\sum_{i=1}^{m}v_{ijd}x_{ij}}.\;d=1,2,\ldots ,n \end{array}$$

The corresponding model is

(14) $$\begin{array}{c} \max\sum_{r=1}^{s}u_{rjd}y_{rj},\\ s.t.\sum_{r=1}^{s}u_{rjd}y_{rj}-\sum_{i=1}^{m}v_{ijd}x_{ij}\leq 0,\\ \sum_{i=1}^{m}v_{ijd}x_{ij}=1,\\ \alpha_{d}\sum_{i=1}^{m}\left(v_{ijd}x_{id}\right)-\sum_{r=1}^{s}\left(u_{rjd}y_{rd}\right)\leq 0,\\ u_{rjd},v_{ijd}\geq 0. \end{array}$$

## 5. Empirical Analysis on Game Cross-Efficiency

### 5.1. Principal Component Analysis (PCA) of Influencing Factors of Rural Revitalization and Urban-Rural Integration

The influencing factors were analyzed with SPSS software. The results of the corresponding total variance explained are shown in Table 3.

The analysis results of the component scoring system matrix for the influencing factors are shown in the following Table 4.

Therefore, its corresponding regression equation is

 
*Z*1 = 0.174 *∗X*1 + 0.228 *∗X*2 + 0.200 *∗X*3 − 0.105 *∗X*4 − 0.170*∗X*5 − 0.115*∗X*6 + 0.200*∗X*7 + 0.084 *∗X*8 − 80.131*∗X*9
 
*Z*2 = −0.303*∗X*1 − 0.096 *∗X*2 − 0.029 *∗X*3 − 0.343*∗X*4 − 0.256*∗X*5 + 0.080*∗X*6 + 0.114 *∗X*7 + 0.501 *∗X*8 + 0.421*∗X*9
 
*Z*3 = 0.345 *∗X*1 + 0.077*∗X*2 + 0.115 *∗X*3 + 0.579 *∗X*4 + 0.236 *∗X*5 − 0.187 *∗X*6 − 0.010*∗X*7 + 0.429*∗X*8 + 0.417*∗X*9.

By the regression variance, we can calculate the results of three principal components of the influencing factors in 16 cities of Anhui Province. The specific condition is shown in Table 5.

### 5.2. Data Envelopment Model Analysis of Influencing Factors of Rural Revitalization and Urban-Rural Integration

The MaxDEA software is used to calculate the above three efficiency values, and the calculation results are shown in Table 6.

By the above calculation results, we can derive a trend chart of efficiency indicators, as shown in Figure 1.

### 5.3. Result Analysis

#### 5.3.1. Regional Development Is Unbalanced, and Echelon Distribution Is Significant

From the efficiency results of 16 cities in Anhui Province, it can be seen that Hefei and Tongling belong to the first echelon; Ma'anshan, Huaibei, Huainan, and Wuhu belong to the second echelon; Bengbu, Xuancheng, Chuzhou, Chizhou, Anqing, and Huangshan belong to the third echelon; and Fuyang, Lu'an, Suzhou, and Bozhou belong to the fourth echelon.

#### 5.3.2. The Results of BCC Efficiency and Cross-Efficiency Are Similar, but There Are Slight Differences

From the comparison of the BCC efficiency and cross-efficiency results of 16 cities in Anhui Province, it can be seen that the ranking of efficiency values that are calculated by the two calculation methods has not almost changed. However, there are slight differences between the two groups of cities: Ma'anshan and Huaibei, and Anqing and Huangshan.

We can learn from the analysis that one of the main reasons for the above situation is that BCC efficiency and cross-efficiency are similar. The BCC efficiency in data envelopment analysis is mainly determined by the way that is most beneficial to the evaluated DMUs, while the cross-efficiency model evaluates all DMUs with each group of weights. In addition, the input and output indexes of Ma'anshan and Huaibei, Anqing and Huangshan are similar, so this is how the above analysis results are similar but slightly different.

#### 5.3.3. Combined with the Analysis of Game Cross-Efficiency, the Differences among Cities in Anhui Province Are Obvious

By combining with the analysis, it is found that the game cross-efficiency of Hefei, Xuancheng, and Huangshan fluctuates with BCC efficiency and cross-efficiency. From the comparison results of 16 cities in Anhui Province, it is found that the efficiency of urban-rural integration in Hefei in the first echelon declines significantly, while that in Huangshan and Xuancheng, the third echelon sees a rising trend, and especially, the rising extent of Huangshan is significant.

It is found from the above analysis that Hefei's attraction to the country is relatively insufficient. Tongling has done a good job in the urban-rural integration, because it is small, with little difference between city and country, and it has fewer difficulties than other cities [17]. Huangshan and Xuancheng have relatively strong competitiveness in potential and attractiveness in the future.

## 6. Conclusion and Suggestions

### 6.1. Strategic Direction of Building an Urban-Rural Integration System

In order to implement the rural revitalization strategy, we should, by taking cities and countries as organic systems, build a coupling model and innovation system that integrates “human,” “land” with “industry” in rural areas to promote gather of capital, talents, and other elements in rural areas, gradually break the urban-rural functional division pattern, and realize urban and rural areas support each other, integrate with each other and make progress simultaneously.

### 6.2. Overall Design of Urban and Rural Functional Planning

A convenient and smooth transportation network system from the market to the field can be formed through the implementation of construction projects. The consolidation and upgrading project of urban and rural basic infrastructure can be implemented to improve and build an efficient network [18]. We should implement the overall design of functional planning, implement informatization construction projects, develop a safe and efficient information and communication network with reasonable urban and rural layout, balanced development and perfect functions, implement the digital rural strategy, and comprehensively promote the “Internet+.”

### 6.3. Promote Cobuilding and Sharing of Urban and Rural Infrastructure

The government should vigorously promote the network infrastructure construction that fits the demands of agriculture, rural areas, and farmers, adhere to overall planning, urban-rural integration, focus on weakness and break major problems, accelerate the upgrading of urban and rural infrastructure, and build a safe, efficient, and connective infrastructure network system [19]. According to local conditions, the government should implement a demonstration pilot project of integrated urban-rural development, promote upgrading and transformation of urban and rural infrastructure to realize joint construction and sharing, and calmly realize the overall goal of building space that is suitable for both living and industry development and picturesque ecological scenery.

## Figures and Tables

**Figure 1:** Trend chart of efficiency indicators.

**Table 1:** Index system of crossover analysis.

	Thriving business	Pleasant living environment	Rural civilization	Effective governance	Living in abundance
Spatial layout	*X*1	—	—	—	—
Industry configuration	*X*2	—	—	*X*3	—
Public service	*X*4	*X*5	*X*6	*X*7	—
Ecological environment	—	*X*7	—	*X*8	—
Income gap	—	—	—	—	*X*9

**Table 2:** General cross-efficiency matrix.

Evaluated units	1	2	3	…	*n*
1	*E*_11_	*E*_12_	*E*_13_	…	*E*_1*n*_
2	*E*_21_	*E*_22_	*E*_23_	…	*E*_2*n*_
3	*E*_31_	*E*_32_	*E*_33_	…	*E*_3*n*_
…	…	…	…	…	…
*n*	*E*_*n*1_	*E*_*n*2_	*E*_*n*3_	…	*E*_*nn*_
Average value	$\bar{E_{1}}$	$\bar{E_{2}}$	$\bar{E_{3}}$	…	$\bar{E_{n}}$

**Table 3:** Total variance explained of influencing factors of rural revitalization and urban-rural integration.

Component	Initial eigenvalue			Loading of quadratic sum extracted		
	Total	Variance	Accumulation	Total	Variance	Accumulation
1	4.175	46.386	46.386	4.175	46.386	46.386
2	1.365	15.164	61.550	1.365	15.164	61.550
3	1.084	12.047	73.597	1.084	12.047	73.597
4	0.876	9.730	83.327			
5	0.631	7.007	90.335			
6	0.406	4.515	94.850			
7	0.219	2.428	97.278			
8	0.202	2.247	99.524			
9	0.043	0.476	100.000			

**Table 4:** Component scoring system matrix for influencing factors.

	Component		
	1	2	3
*X*1 ratio of nonagricultural workers to agricultural workers	0.174	−0.303	0.345
*X*2 ratio of nonagricultural output value to agricultural output value	0.228	−0.096	0.077
*X*3 ratio of hospital bed in city and hospital bed in country (%)	0.200	−0.029	0.115
*X*4 air quality reaching or better than grade II (%)	−0.105	−0.343	0.579
*X*5 green coverage ratio of built-up area (%)	−0.170	−0.256	0.236
*X*6 ratio of urban subsistence allowance per capita and rural subsistence allowance per capita (%)	−0.115	0.080	−0.187
*X*7 ratio of urban middle school enrollment to rural middle school enrollment (%)	0.200	0.114	−0.010
*X*8 ratio of urban sewage treatment to rural sewage treatment (%)	0.084	0.501	0.429
*X*9 ratio of disposable income in rural towns	−0.131	0.421	0.417

**Table 5:** Calculation of the three principal components of influencing factors.

No.	City	Input variable			Output variable
		Principal component 1	Principal component 2	Principal component 3	
1	Hefei	2.92	35.55	102.66	76.33
2	Huaibei	15.00	24.41	107.22	65.88
3	Bozhou	27.96	26.91	113.56	42.22
4	Suzhou	25.73	22.45	112.68	43.96
5	Bengbu	23.10	16.24	124.91	58.58
6	Fuyang	22.88	26.29	107.68	44.62
7	Huainan	16.26	25.31	106.35	65.04
8	Chuzhou	16.38	21.00	117.36	54.54
9	Lu'an	25.64	15.55	125.85	47.09
10	Ma'anshan	6.64	30.74	106.02	69.12
11	Wuhu	8.24	32.36	113.30	66.41
12	Xuancheng	11.98	16.20	125.09	56.33
13	Tongling	5.91	2.06	101.12	57.16
14	Chizhou	15.69	18.58	125.60	54.92
15	Anqing	18.59	20.37	117.78	49.98
16	Huangshan	11.04	12.10	133.12	52.49

**Table 6:** Calculation and ranking of efficiency of rural revitalization and urban-rural integration.

No.	City	BCC model	Ranking	Cross-efficiency model	Ranking	Game cross-efficiency model	Ranking
1	Hefei	1.00	1	0.94	1	0.20	5
2	Tongling	1.00	1	0.96	2	0.49	1
3	Ma'anshan	0.91	3	0.83	3	0.20	5
4	Huaibei	0.91	3	0.81	4	0.21	4
5	Huainan	0.89	5	0.80	5	0.20	5
6	Wuhu	0.83	6	0.75	6	0.18	9
7	Bengbu	0.75	7	0.67	7	0.17	11
8	Xuancheng	0.72	8	0.65	8	0.23	3
9	Chuzhou	0.71	9	0.64	9	0.18	9
10	Chizhou	0.69	10	0.62	10	0.19	8
11	Anqing	0.65	11	0.58	11	0.16	12
12	Huangshan	0.65	11	0.59	12	0.25	2
13	Fuyang	0.60	13	0.54	13	0.12	14
14	Lu'an	0.60	13	0.54	13	0.13	13
15	Suzhou	0.59	15	0.52	15	0.12	14
16	Bozhou	0.54	16	0.48	16	0.11	16

## Data Availability

The data used to support the findings of this study are included within the article.
